# A Novel-Defined Necroptosis-Related miRNA Signature for Forecasting the Prognosis of Low-Grade Glioma

**DOI:** 10.1155/2022/9957604

**Published:** 2022-09-25

**Authors:** Zhuangzhuang Lu, Chao Wang, Tingting Qu, Yugong Feng

**Affiliations:** ^1^Department of Neurosurgery, The Affiliated Hospital of Qingdao University, Qingdao City 266000, China; ^2^Department of Pathology, The Affiliated Hospital of Qingdao University, Qingdao City 266000, China

## Abstract

**Background:**

Increasing evidence has shown that necroptosis has enormous significance in the generation and deterioration of cancer, and miRNA molecular markers involved in necroptosis in low-grade gliomas (LGGs) have not been thoroughly reported.

**Methods:**

Using the miRNA data of 512 samples from The Cancer Genome Atlas (TCGA), 689 miRNAs from LGG samples were split into high immunity score and low immunity score groups for analysis. The differential miRNAs related to necroptosis were analyzed by univariate Cox regression analysis. On the basis of the outcome of univariate Cox regression analysis, miRNAs with significant differences were selected to construct a multivariate Cox regression model and calculate the risk score. Then, we evaluated whether the risk score could be used as an unaided prognostic factor.

**Results:**

Overall, six differential miRNAs were identified (*hsa-miR-148a-3p*, *hsa-miR-141-3p*, *hsa-miR-223-3p*, *hsa-miR-7-5p*, *hsa-miR-500a-3p*, and *hsa-miR-200a-5p*). Univariate and multivariate Cox regression analyses were performed, and the *c* index was 0.71. Then, by mixing the risk score with clinicopathological factors, univariate Cox regression (HR: 2.7146, 95% CI: 1.8402−4.0044, *P* < 0.0001) and multivariate Cox regression analyses (HR: 2.3280, 95% CI: 1.5692−3.4536, *P* < 0.001) were performed. The data suggested that the risk score is an unaided prognostic indicator, which is markedly related with the overall survival time of LGG sufferers. Thus, a lower risk score is correlated with better prediction of LGG.

**Conclusion:**

In order to achieve the ultimate goal of improving the living conditions of patients, we established prognostic risk model using 6 miRNAs related to necroptosis, which has the ability to predict the prognosis of LGG. It is possible to further enrich the therapeutic targets for LGG and provide clinical guidance for the treatment of LGG in the future.

## 1. Introduction

Pathologically, gliomas can be divided into oligodendrogliomas, astrocytomas, and mixed oligodendrogliomas [1]. LGGs are gliomas, accounting for approximately 20% of total brain malignant pathological changes. They grow slowly and have a survival time of 5-10 years. The following are the high-danger elements for the progression of LGG to high-grade gliomas: preoperative neurological dysfunction, age over 40 years, tumor diameter ≥ 6 cm, and tumor traversing the midline [2]. New molecular indicators, including *p53* mutation, isocitrate dehydrogenase 1 (*IDH1*) mutation, and 1p/19q chromosomal codeletion, have been found to improve the treatment status and overall survival time of LGG [3]. However, at present, few molecular signatures have been recognized to predict the clinical quality of life of glioma cases. Therefore, in-depth exploration of the pathogenic mechanism of LGGs is very important to find new treatment and prognostic targets for LGGs.

Necroptosis is a method of programmed cell death that plays an important role in tumor biology, including tumor transmutation, subtypes, and immunity [4]. Necroptosis is a mixture of apoptosis and necrosis with a binary function in tumors. First, it has been confirmed that key necroptotic molecules promote tumor progress [5]. In contrast, necroptosis is a mechanism to prevent the development of cancer [6]. It has been reported that the production of key indicators of necroptosis is widely downregulated in tumors. A variety of therapeutic drugs can treat and prevent cancer by regulating the molecular mechanism of necroptosis. Considering the key effect of necroptosis on tumor pathophysiology, it has become a novel marker for the prediction and treatment of cancer. Current study has shown that the induction of necroptosis has become a way to cure drug-resistant tumors [7]. Some researchers [8] have used bioinformatics methods to point out that the high expression of receptor interacting protein kinasess1 and 3 (*RIPK1* and *RIPK3*) and multiple-lineage-like kinase (*MLKL*) related to necroptosis are negative prognostic indicators of LGG. Another literature reported that the analysis of *RIPK3* expression level and isocitrate dehydrogenase (IDH) mutation state together can improve the overall survival rate of LGG [9].

MicroRNAs (miRNAs) are endosomal noncoding RNAs that silence protein-coding genes by binding with the 3′-untranslated region of related mRNA, thus giving rise to separation of those mRNAs or suppressing their translation [10]. Thus, miRNAs act as specific factors in posttranscriptional gene silencing. miRNAs participate in many biological processes and are critical indicators of cell germination and homeostasis. These tiny RNAs affect the production of a variety of proteins by regulating the target mRNA and play a key role in cell behavior. Therefore, miRNA dysfunction may lead to disease. Studies have found differentially regulated miRNAs in many types of cancer, involving pathophysiological activities, such as tumor cell generation, proliferation, migration, and regulation, to guide the development or inhibition of cancer [11]. Many studies have shown that miRNAs affect the production and development of LGG; for example, *Hoxa-AS2*, as the ceRNA of *miR-184*, regulates the production of *COL6A2* and then induces the growth and proliferation of LGG cells [12]. However, there are no specific studies on the use of necroptosis-related miRNAs to predict the survival status of LGG cases. Therefore, it is unclear whether necroptosis-related miRNAs are related to the prognosis of LGG patients, and it is necessary to explore the use of necroptosis-related miRNAs to anticipate the survival of LGG patients.

To address the above problem, this study first downloaded the public database of LGG miRNA expression data and related clinical data and extracted necroptosis-related miRNA data. Then, prognostic molecular markers were constructed by difference analysis and univariate and multivariate Cox regression model analyses. This study describes the correlation between miRNAs and clinical factors and immune cells. Finally, the target genes and lncRNAs related to the most conspicuous prognostic miRNAs were predicted, and miRNA and target genes as well as lncRNA networks were established. Functional enrichment analysis of the interrelated genes was executed to probe the potential pathways of these miRNAs.

## 2. Materials and Methods

### 2.1. Data Collection and Sample Extraction

In our research, miRNA expression data and related clinical factor data of LGG cases were obtained from the TCGA database (https://portal.gdc.cancer.gov/). The inclusion criteria were as follows: (1) patients diagnosed with LGG and (2) patients who had complete miRNA and clinical data. Among them, there were 512 samples of miRNA data and 511 samples of clinical data. The immune score of LGG was searched from ESTIMATE (http://bioinformatics.mdanderson.org/estimate/). In this research, all samples were required to have immune scores [13]. Because the median immune score was the cutoff criterion, this study included 689 miRNAs from LGG samples to divide them into high and low immune score groups. Considering that the data were from the TCGA database and strictly followed the TCGA publication guidelines (http://cancergenome.nih.gov/abouttcga/policies/publicationguidelines), the consent of the Ethics Committee was not needed.

### 2.2. Screening of miRNAs Related to Necroptosis

The following necroptosis miRNAs related to cancer development were collected from the literature [14]: *miR-495*, *miR-331-3p*, *miR-15a*, *miR-148a-3p*, *miR-7-5p*, *miR-141-3p*, *miR-425-5p*, *miR-200a-5p*, *miR-210*, *miR-223-3p*, *miR-500a-3p*, *miR-181-5p*, and *miR-16-5p*. Then, a miRNA expression matrix related to necroptosis was extracted. We also carried out data matching, filtering, and correction, as well as filtering and matching the relevant clinical data for the use of follow-up analysis.

### 2.3. Construction of the miRNA Prognostic Model Related to Necroptosis

In this study, the “limma” package of R software was utilized to analyze differences in the processed data. The filtering conditions were as follows: the absolute value of log2FC was greater than 0.5 and FDR < 0.05. The necroptosis miRNAs meeting the above filtering conditions were considered to be differentially expressed. The differentially expressed miRNAs related to necroptosis were analyzed by univariate Cox regression analysis. On the basis of the outcome of univariate Cox regression analysis, the significantly differentially expressed miRNAs associated with necroptosis were selected to construct a multivariate Cox regression model and obtain the risk score. In addition, the risk score acquired by the model was combined with clinical factors for univariate Cox regression analysis and multivariate Cox regression analysis to determine whether the risk score could be an absolute prognostic indicator. In this study, the predictive ability of the model was evaluated by drawing ROC curves to calculate the AUC. The risk score is calculated based on the normalized expression level of each genes and the corresponding regression coefficient. The formula is as follows: *Risk* *Score* = (*X* : coefficients, *Y* : gene expression level). In line with the median risk score, the data were split into low- and high-risk groups, and the survival curve related to the risk score was drawn. To further clarify the clinical correlation between these significant miRNAs and LGG patients, the survival curve of each miRNA in the model was drawn in batches to obtain clearly differentially expressed miRNAs (*P* < 0.05).

### 2.4. The Correlation between Significant miRNAs in the Prognosis of LGG and Clinical Factors

We also used the Mann–Whitney *U* test statistical method to determine the relevance of clinical factors (age, race, sex, tumor grade, pathology, isocitrate dehydrogenase (IDH) status, 1p/19q codeletion, disease-specific survival event (DSS event), laterality, overall survival (OS), progression-free interval event (PFI event), and primary therapy outcome) and significant differentially expressed miRNAs in the prognosis of LGG. “ggplot2” was the main R package used to visualize the data. The miRNAseq data (in mapped reads per million) were transformed into log2 format, the control/normal data were removed (not all items had control/normal data), the clinical information was retained, and the corresponding box diagram was drawn. The coxph function of R language, the statistical methods of Wald test and score (log-rank) test, and the likelihood ratio test were used to analyze the Cox regression of single and multiple factors. Significant miRNAs were also used to draw ROC curves to calculate 1-year, 3-year, and 5-year AUCs for LGGs. We used the chi-squared statistical method to combine the most predictive miRNAs in the ROC curve with clinical factors and then drew the relevant baseline data table. The univariate logistic regression analysis table related to clinical factors of the most predictive miRNAs was calculated by using a binary logistics model, as well as the subgroup analysis.

### 2.5. The Correlation between the Most Predictive miRNAs and Immunity

The ssGSEA algorithm and Spearman correlation analysis were used to analyze the most predictive miRNAs and 24 types of immune cells (NK CD56dim cells; natural killer (NK) cells; NK CD56bright cells; macrophages; immature DCs (iDCs); eosinophils; cytotoxic cells; cytotoxic cells; CD8 T cells; T helper 17 (Th17) cells; B cells; T helper 2 (Th2) cells; activated DCs (aD); and regulatory cells (Tregs)) and their infiltration relationships using the “GSVA” package and to draw the corresponding lollipop diagram and scatter plot.

### 2.6. Network and Enrichment Analysis of Target Genes

Three databases, TargetScan (http://www.targetscan.org/vert_71/), miRDB (http://mirdb.org/), and miTarBase (http://miRTarBase.cuhk.edu.cn/), were used to identify the target genes of necroptosis-related miRNAs significantly related to prognosis. Meanwhile, the target genes of necroptosis-related miRNAs had to exist in all three databases. Cytoscape software was used to draw a miRNA-target gene meshwork, and the R package “clusterProfiler” was used to identify Gene Ontology (GO) and the Kyoto Encyclopedia of Genes and Genomes (KEGG) pathways. We also predicted lncRNAs by miRNAs through the starBase (http://starbase.sysu.edu.cn/) website and established the corresponding network diagram through the predicted lncRNAs.

### 2.7. Statistical Analysis

The Kaplan-Meier statistical approach was used for survival curves, and the logarithmic rank test was applied for comparisons. Evaluation of the miRNA signature related to necroptosis by Cox regression, the effect of risk score and clinicopathological data on prognosis, and the Mann–Whitney *U* test statistical approach were utilized to assess the relationship between miRNA and clinical factors. The baseline data table of miRNAs related to clinical factors was calculated by the chi-squared test, and the univariate logistic regression analysis table was calculated by a binary logistics model. The most predictive miRNAs and 24 types of immune cells were determined by Spearman correlation analysis. R language (version 4.1) was used to perform the statistical calculations. Statistical significance was indicated as follows: ns, *P* ≥ 0.05; ^∗^, *P* < 0.05; ^∗∗^, *P* < 0.01; ^∗∗∗^, *P* < 0.001.

## 3. Results

### 3.1. Results of the miRNA Prognostic Model Related to Necroptosis

According to the results of difference analysis, 6 differentially expressed miRNAs were obtained: hsa-miR-200a-5p, hsa-miR-148a-3p, hsa-miR-223-3p, hsa-miR-500a-3p, hsa-miR-141-3p, and hsa-miR-7-5p (Figure 1). Therefore, we selected the above 6 miRNAs to construct a univariate Cox regression model (Figure 2(a)) and multivariate Cox regression model (Figure 2(b)). The *C* index of the prediction model was 0.71. The risk score was calculated as follows: Risk Score = (0.19715∗hsa − miR − 141 − 3p exp.) + (1.22675∗hsa − miR − 148a − 3p exp.) + (0.50959∗hsa − miR − 200a − 5p exp.) + (0.19281∗hsa − miR − 223 − 3p exp.) + (−0.53776∗hsa − miR − 500a − 3p exp.) + (−0.01312∗hsa − miR − 7 − 5p exp.). The risk score was computed and then combined with clinical factors for univariate and multivariate Cox regression analyses (univariate Cox regression: HR: 2.7146, 95% CI: 1.8402-4.0044, *P* < 0.0001, Figure 2(c); multivariate Cox regression: HR: 2.3280, 95% CI: 1.5692-3.4536, *P* < 0.001, Figure 2(d)). The results indicated that the risk score of this model could be an absolute prognostic indicator and significantly correlated with the total OS of LGG cases. Meanwhile, the outcome of the survival curve drawn in accordance with the risk score also certified that the low risk score had a better prognosis for LGGs (*P* < 0.001, Figure 2(e)). The outcome of the ROC curve shows that the model had a certain predictive ability (Figure 2(f)). The areas under the ROC curve of 1-year, 3-year, and 5-year survival were 0.8, 0.667, and 0.721, respectively. To further identify the necroptosis miRNAs that predict LGGs, we conducted a batch of survival analysis of miRNAs and found that *hsa-miR-141-3p* (*P* = 0.00087), *hsa-miR-148a-3p* (*P* < 0.001), *hsa-miR-200a-5p* (*P* < 0.001), *hsa-miR-223-3p* (*P* = 0.02081), and *hsa-miR-500a-3p* (*P* = 0.01373) were markedly related with the survival state of LGGs, with higher expression correlating with worse prognosis (Figure 3).

### 3.2. Correlation between miRNAs That Are Markedly Related to the Prognosis of LGG and Clinical Factors

The Mann–Whitney *U* test was performed to estimate the associations between *hsa-miR-200a-5p*, *hsa-miR-148a-3p*, *hsa-miR-223-3p*, *hsa-miR-141-3p*, and *hsa-miR-500a-3p* expression and 12 clinicopathological variables, including age, race, sex, tumor grade, pathology, IDH status, 1p/19q codeletion, DSS event, laterality, OS, PFI event, and primary therapy outcome. The results are shown in Figure 4.

Univariate and multivariate Cox risk regression analyses were performed to screen absolute prognostic indicators from *hsa-miR-200a-5p*, *hsa-miR-148a-3p*, *hsa-miR-223-3p*, *hsa-miR-141-3p*, *hsa-miR-500a-3p*, race, WHO grade, histological type, 1p/19q codeletion, age, gender, IDH status, laterality, and primary therapy outcome. Univariate Cox risk regression analysis demonstrated that *hsa-miR-141-3p* grade, primary therapy outcome, age, 1p/19q codeletion, and IDH status were significantly correlated with OS (*P* < 0.05). Multivariate Cox risk regression analysis demonstrated that *hsa-miR-500a-3p*, *hsa-miR-148a-3p*, WHO grade, age, sex, IDH status, and primary therapy outcome were markedly related with OS (*P* < 0.05) (Table 1).

We also drew ROC curves of the 5 significant miRNAs in LGG and calculated the AUC, as shown in Figure 5. Among them, *hsa-miR-148a-3p* (1-year (AUC = 0.825); 3-year (AUC = 0.712); 5-year (AUC = 0.670)) and *hsa-miR-200a-5p* (1-year (AUC = 0.771); 3-year (AUC = 0.680); 5-year (AUC = 0.651)) had better predictive results.

We summarized the correlation between the 2 miRNAs and clinical parameters (sex, 1p/19q codeletion, histological type, age, IDH status, laterality, WHO grade, primary therapy outcome, OS event, DSS event, PFI event, and race). The 2 miRNAs were separated into high expression and low expression in clinical parameters and then analyzed by modified Fisher's test (Tables 2 and 3). The clinical parameters of the 2 miRNAs (IDH status, sex, primary therapy outcome, 1p/19q codeletion, WHO grade, and age) were analyzed by univariate logistic analysis: *hsa-miR-148a-3p* and primary therapy outcome, IDH status, and 1p/19q codeletion had significant meaning (Table 4); and *hsa-miR-200a-5p* and 1p/19q codeletion, age, and IDH status had significant meaning (Table 5). Then, we performed a subgroup analysis of the 2 miRNAs in terms of age, sex, and WHO grade: the 2 miRNAs confirmed that the low-expression group was better than the high-expression group in terms of OS (Figure 6), but age: ≤40 and WHO grade: G2 of *hsa-miR-148a-3p* did not show significance.

### 3.3. Correlation between miRNA and Immunity in Patients with LGGs

Immune infiltration algorithm: ssGSEA (GSVA package) and Spearman correlation analysis were applied to analyze the relationship between *hsa-miR-148a-3p*, *hsa-miR-200a-5p*, and 24 types of immune cells, and an immune-related lollipop map (Figure 7) and the related scatter plot were drawn (Figures 8 and 9). The range of correlation coefficient *r* is −1 ≤ *r* ≤ 1. Negative values represent negative correlation, and positive values represent positive correlation. There was no significant correlation between *hsa-miR-200a-5p* and *hsa-miR-148a-3p* and DC, Tcm, Tem, and Th2 cells or Treg in LGG. Moreover, *hsa-miR-148a-3p* and T helper cells had no clear relationship.

### 3.4. Outcome of Enrichment Analysis of Target Genes

*Hsa-miR-148a-3p* and *hsa-miR-200a-5p*, which were markedly correlated with the prognosis of LGG, were chosen to predict target genes, and 79 target genes were obtained (Figure 10(a)). A meshwork diagram of the interaction between miRNA and target genes was constructed by Cytoscape software, as shown in Figure 10(b). Finally, the 79 target genes were analyzed by GO and KEGG enrichment analysis. The outcome of GO enrichment analysis revealed that these target genes were significantly enriched as follows: cardiac muscle tissue development function, mesenchyme morphogenesis, organ growth, cardiac muscle tissue growth, and phagolysosome assembly (Figure 10(c)) (only the first five most significant pathways are listed here). The results of KEGG enrichment analysis showed that these target genes were associated with miRNAs in cancer, hepatocellular carcinoma, signaling pathways regulating pluripotency of stem cells pathways, the *FoxO* signaling pathway, and proteoglycans in cancer (Figure 10(d)) (only the first five most significant pathways are listed here), which means that *hsa-miR-200a-5p* and *hsa-miR-148a-3p* are related to these functions and pathways.

We predicted *hsa-miR-148a-3p*-related lncRNAs through the website, obtained 25 related lncRNAs, and used Cytoscape software to draw the relevant targeted network diagram (Figure 10(e)). This will promote our understanding of the molecular pathways of *hsa-miR-148a-3p* involved in necroptosis in LGG and may provide ideas for finding new therapeutic targets in the future.

## 4. Discussion

Programmed cell death (PCD) is defined as regulatory cell death during the execution of intracellular programs. Traditionally, apoptosis is considered the sole format of programmed cell death. However, in recent years, it has also included necroptosis, which has become a natural barrier to limit the survival and spread of malignant cells. Necroptosis plays a key role in immune monitoring, subtype, prognosis, and progress of cancer patients [15]. miRNAs regulate approximately 50% of protein-coding genes and have considerable effects in almost all kinds of biological events. Many miRNAs are able to strongly regulate the output of proapoptosis and antiapoptosis genes, necroptosis-related genes, endoplasmic reticulum stress, and oncogenes [16]. Changes in miRNA expression are related with the occurrence and survival outcome of non-small-cell lung cancer [17]. *MiRNA-221* is upregulated in glioblastoma and regulates inhibition of the tumor gene *p27* [18]. In contrast, epidermal growth factor receptor is regulated by downregulating *miR-7* to decrease the proliferation and invasiveness of cultured glioma cells [19]. Many studies have proven that miRNAs can regulate the prognosis of gliomas, suggesting that miRNAs can be used as latent markers for the survival of gliomas. Therefore, it is necessary to establish a miRNA signature related to necroptosis on the basis of a large database to predict the survival outcomes of patients with LGGs.

Although many studies have used miRNAs as molecular markers to predict the survival of tumor patients, there are no studies on the systematic use of necroptosis-related miRNAs to predict survival of LGG. Our research probes the use of necroptosis-related miRNAs to predict the survival outcome of patients with LGGs for the first time. In our research, we collected necroptosis-related miRNAs related to cancer development from the literature [14]. Then, 6 miRNAs were selected to construct models by difference analysis. On the basis of the outcome of the *C* index and ROC curve, the model had better differentiation and accuracy, and the OS of the high-risk group was shorter than that of the low-risk group. The areas under the ROC curve of 1-year, 3-year, and 5-year survival were 0.8, 0.667, and 0.721, respectively. Among them, *hsa-miR-500a-3p*, *hsa-miR-148a-3p*, *hsa-miR-223-3p*, *hsa-miR-200a-5p*, and *hsa-miR-141-3p* were markedly related with the survival outcome of LGGs, which may be highly related with the generation and evolution of LGGs.

Five necroptosis-related miRNAs (*hsa-miR-141-3p*, *hsa-miR-148a-3p*, *hsa-miR-200a-5p*, *hsa-miR-223-3p*, and *hsa-miR-500a-3p*) were found to be related to tumors. (1) *ZEB2* is regulated by *hsa-miR141-3p*, and its expression is markedly decreased in some gastric adenocarcinoma brain metastases [20]. Moreover, studies have confirmed that *hsa-miR-141-3p* has a key effect on the regulation of miRNA in bladder tumors [21]. (2) Access to *miR-148a-3p/ERBB3/AKT2/c-myc* signaling plays a key role in regulating the evolution of bladder tumors. Moreover, research has found that *MYC* is a target gene of *miR-148a*, whose expression is decreased in gastric cancer [22]. We believe that *miR-148a-3p* participates in the progression of gastric cancer by regulating *MYC* [23]. (3) *MiR-200a-5p* has an enormous role in distinguishing between nonmalignant thyroid tumors and papillary thyroid carcinoma [24]. (4) *hsa-miR-223-3p* participates in the growth and invasion of cancer [25]. *Hsa-miR-223-3p* is a marker to predict the survival of patients with kidney renal clear cell carcinoma [26]. *MiR-223-3p* has a carcinogenic effect in colon tumors by regulating *EMT* and *PRDM1* [27]. (5) *MiR-500a-3P* appears to be effective in endometriosis, hepatocellular carcinoma, and breast cancer [28–30]. A previous study also demonstrated that *miR-500* results in gastric tumor cell progression while preventing apoptosis [31].

No miRNA molecular marker has been proven to be effective in adjuvant chemotherapy or radiotherapy in LGG, which provides a basis for molecular therapy in the treatment of LGG in the future [32]. Through survival analysis of miRNAs in the model, 5 miRNAs were markedly related with the prognosis of LGGs, and the correlation with clinical factors was then analyzed. According to univariate and multivariate Cox risk regression analyses, *hsa-miR-148a-3p*, IDH status, age, primary therapy outcome, and WHO grade were all independent prognostic indicators of LGG.

Moreover, we drew the ROC curves of 5 significant miRNAs in LGG and calculated the AUC. *Hsa-miR-200a-5p* and *hsa-miR-148a-3p* had the strongest predictive effect. Furthermore, the correlation between the 2 miRNAs and clinical parameters was analyzed; univariate logistic analysis and subgroup analysis with age, sex, and WHO grade were carried out; and it was concluded that the OS in the high-expression group was worse than that in the low-expression group.

Necroptosis participates in tumor-relevant immune reactions, which promote the relationship between moribund tumor cells and immune cells through cytokines and chemokines within the tumor microenvironment [33]. We used the ssGSEA algorithm to analyze the correlation between *hsa-miR-200a-5p*, *hsa-miR-148a-3p*, and 24 types of immune cells. In LGG, *hsa-miR-200a-5p* and *hsa-miR-148a-3p* are associated with a large number of immune cells, indicating that these 2 molecules are likely to be immune-related markers of necroptosis in tumors.

A study proposed that necroptosis-related genes are involved in the formation of tumor immune microenvironment and can recruit immune cells to promote the proliferation of cancer cells [34]. For example, *RIPK3* is involved in regulating the expression of cytokines in DC, and DC is the key cell that regulates the dynamic balance of the immune system [35]. Therefore, to explore the relationship between necroptosis-related miRNAs and immune cells is to better understand the mechanism of action of necroptosis-related miRNAs in tumor, which has guiding significance for the study of necroptosis-related antineoplastic drugs.

The results of enrichment analysis showed that these miRNAs related to necroptosis were markedly enriched in tumor-related pathways and other biological processes. For example, in KEGG analysis, *hsa-miR-200a-5p* and *hsa-miR-148a-3p* were mainly enriched in miRNAs in tumors, hepatocellular carcinoma, and proteoglycans in cancer. *MiR-148a-3p* is a key regulator that participates in the progression of many cancers. Overexpression of *miR-148a* restrains the development of breast cancer cells by regulating *WNT-1*, but *miR-148a-3P* has an adverse role [36]. *Hsa-miR-200a-5p* is highly expressed in esophageal adenocarcinoma, pancreatic cancer, colorectal cancer, and other tumors. *Hsa-miR-200a-5p* is expressed in thyroid nonmalignant cancer and thyroid papillary carcinoma [24].

Molecular types of LGG has been paid more and more attention, such as IDH mutation, 1p/19q codeletion, MGMT promoter methylation, and TERT promoter mutation. But all of them have a certain false-positive rate or false-negative rate. LGG is heterogeneous, and finding a stable and controllable target can affect the metabolic renewal and developmental plasticity of cancer cells, which can fundamentally solve the situation of poor prognosis of patients. Our study established a necroptosis-related prognostic model for LGG. Our results suggest that the model plays a good role in evaluating the survival rate of LGG, and the *hsa-miR-200a-5p* and *hsa-miR-148a-3p* with good prognostic ability in the model is closely related to clinicopathological factors. Moreover, the expression of *hsa-miR-200a-5p* and *hsa-miR-148a-3p* regulates immune cells, which may be related to the formation of tumor immunosuppressive microenvironment and immune escape and play a role in tumor microenvironment. To sum up, the prognostic model established by 6 necroptosis-related miRNAs in LGG is a promising prognostic model in LGG, and *hsa-miR-200a-5p* and *hsa-miR-148a-3p* can be used as prognostic markers.

This study only used data from the public database TCGA to build the model and did not meet the conditions to collect clinical data for model verification, which is one of the limitations of our study. In addition, we did not have experimental conditions to verify the expression, function, or mechanism of these miRNAs, which are other limitations of our study. We did not find other online databases to verify our findings, and our samples are small, and the results have some limitations. Although we have explored the biological process of *hsa-miR-200a-5p* and *hsa-miR-148a-3p* in LGG, we have not further analyzed the detailed mechanism in LGG.

In summary, our study shows that necroptosis is closely related to LGGs because of the difference in miRNA expression between the low and high immune score groups of LGG. In addition, our 6 necroptosis-related miRNA models can be used as independent prognostic molecular markers for LGGs. By further connecting clinical factors and immune infiltration, the clinical significance of miRNAs as molecular markers in predicting the prognosis of LGGs was discussed. The network established by targeting genes and lncRNAs provides a way to study the pathway of necroptosis-related LGGs in the future. Our research identified a number of late miRNA markers for predicting the survival status of patients with LGGs and established a considerable basis for the discovery of more necroptosis-related genes in the future.

## Figures and Tables

**Figure 1:** Heatmap of differential miRNAs related to necroptosis based on high and low immune scores in LGG.

**Figure 2:** (a) Univariate cox regression model with 6 differential miRNAs; (b) multivariate cox regression model with 6 differential miRNAs; (c) univariate cox regression about risk score and clinical factors; (d) multivariate cox regression about risk score and clinical factors; (e) survival curve drawn according to high and low risk score; (f) ROC curve drawn according to the prediction model.

**Figure 3:** Survival analysis of each significant miRNA (*P* < 0.05).

**Figure 4:** A box diagram drawn from 5 significantly differential miRNAs and clinicopathological factors.

**Figure 5:** ROC curves of 5 significant miRNAs in LGG are drawn, and the AUC area is calculated, respectively.

**Figure 6:** Subgroup analysis of age, sex, and WHO grade about miRNAs, which has the strongest predictive ability.

**Figure 7:** A lollipop map of the correlation between 24 kinds of immune cells and miRNAs, which has the best predictive ability.

**Figure 8:** Scatter plot about *hsa-miR-148a-3p* and 24 types of immune cells.

**Figure 9:** Scatter plot about *hsa-miR-200a-5p* and 24 types of immune cells.

**Figure 10:** (a) The Venn diagram of the target gene predicted by 2 miRNAs with the strongest predictive ability; (b) network diagram of the interaction between miRNAs and target genes; (c) GO enrichment analysis of target genes; (d) KEGG enrichment analysis of target genes; (e) network diagram of the lncRNAs targeted by hsa-miR-148a-3p.

**Table 1:** Univariate and multivariate Cox regression of 5 significant differentially expressed miRNAs and clinical factors.

Characteristics	Total (*N*)	Univariate analysis		Multivariate analysis	
		Hazard ratio (95% CI)	*P* value	Hazard ratio (95% CI)	*P* value
*hsa-miR-141-3p*	528	1.665 (1.326-2.091)	<0.001	1.281 (0.949-1.730)	0.106
*hsa-miR-148a-3p*	528	1.394 (1.268-1.532)	<0.001	1.225 (1.022-1.467)	0.028
*hsa-miR-200a-5p*	528	1.835 (1.506-2.236)	<0.001	1.064 (0.769-1.473)	0.706
*hsa-miR-223-3p*	528	1.199 (1.054-1.365)	0.006	1.006 (0.843-1.201)	0.946
*hsa-miR-500a-3p*	528	1.186 (0.972-1.448)	0.093	0.749 (0.579-0.968)	0.027
WHO grade	466				
G2	220	Reference			
G3	246	3.032 (2.020-4.551)	<0.001	1.929 (1.182-3.148)	0.009
Age	528				
≤40	264	Reference			
>40	264	2.888 (2.004-4.162)	<0.001	2.960 (1.802-4.861)	<0.001
Gender	528				
Female	240	Reference			
Male	288	1.121 (0.797-1.577)	0.512		
IDH status	525				
WT	97	Reference			
Mut	428	0.182 (0.128-0.260)	<0.001	0.463 (0.225-0.954)	0.037
1p/19q codeletion	528				
Codel	171	Reference			
Noncodel	357	2.488 (1.586-3.904)	<0.001	0.944 (0.484-1.840)	0.865
Primary therapy outcome	458				
PD	110	Reference			
SD	148	0.428 (0.283-0.648)	<0.001	0.361 (0.213-0.611)	<0.001
PR	63	0.172 (0.075-0.397)	<0.001	0.171 (0.060-0.484)	<0.001
CR	137	0.119 (0.055-0.260)	<0.001	0.151 (0.067-0.341)	<0.001
Race	517				
Asian	8	Reference			
Black or African American	22	4849148.928 (0.000-Inf)	0.993		
White	487	3285138.716 (0.000-Inf)	0.993		
Histological type	528				
Astrocytoma	196	Reference			
Oligoastrocytoma	133	0.652 (0.413-1.029)	0.066	1.524 (0.860-2.699)	0.149
Oligodendroglioma	199	0.582 (0.396-0.855)	0.006	0.643 (0.351-1.176)	0.152
Laterality	523				
Left	257	Reference			
Midline	7	1.033 (0.312-3.425)	0.958		
Right	259	0.780 (0.549-1.108)	0.165		

Annotation: WT: wild type; Mut: mutation; PD: progress disease; SD: stable disease; PR: partial response; CR: complete response.

**Table 2:** Modified Fisher test of *hsa-miR-148a-3p* and clinical parameters.

Characteristic	Low expression of *hsa-miR-148a-3p*	High expression of *hsa-miR-148a-3p*	*P*
*n*	264	265	
WHO grade, *n* (%)			0.629
G2	111 (23.8%)	110 (23.6%)	
G3	117 (25.1%)	129 (27.6%)	
IDH status, *n* (%)			<0.001
WT	5 (1%)	92 (17.5%)	
Mut	257 (48.9%)	172 (32.7%)	
1p/19q codeletion, *n* (%)			<0.001
Codel	114 (21.6%)	58 (11%)	
Noncodel	150 (28.4%)	207 (39.1%)	
Primary therapy outcome, *n* (%)			0.012
PD	42 (9.2%)	68 (14.8%)	
SD	80 (17.4%)	68 (14.8%)	
PR	37 (8.1%)	26 (5.7%)	
CR	78 (17%)	60 (13.1%)	
Gender, *n* (%)			0.405
Female	115 (21.7%)	126 (23.8%)	
Male	149 (28.2%)	139 (26.3%)	
Race, *n* (%)			0.369
Asian	6 (1.2%)	2 (0.4%)	
Black or African American	10 (1.9%)	12 (2.3%)	
White	242 (46.7%)	246 (47.5%)	
Age, *n* (%)			0.828
≤40	130 (24.6%)	134 (25.3%)	
>40	134 (25.3%)	131 (24.8%)	
Histological type, *n* (%)			0.014
Astrocytoma	83 (15.7%)	113 (21.4%)	
Oligoastrocytoma	67 (12.7%)	66 (12.5%)	
Oligodendroglioma	114 (21.6%)	86 (16.3%)	
Laterality, *n* (%)			0.392
Left	135 (25.8%)	122 (23.3%)	
Midline	3 (0.6%)	4 (0.8%)	
Right	122 (23.3%)	138 (26.3%)	
OS event, *n* (%)			<0.001
Alive	217 (41%)	177 (33.5%)	
Dead	47 (8.9%)	88 (16.6%)	
DSS event, *n* (%)			<0.001
Alive	220 (42.2%)	179 (34.4%)	
Dead	41 (7.9%)	81 (15.5%)	
PFI event, *n* (%)			0.003
Alive	177 (33.5%)	143 (27%)	
Dead	87 (16.4%)	122 (23.1%)	

Annotation: DSS: disease-specific survival; PFI: disease-free interval.

**Table 3:** Modified Fisher test of *hsa-miR-200a-5p* and clinical parameters.

Characteristic	Low expression of *hsa-miR-200a-5p*	High expression of *hsa-miR-200a-5p*	*P*
*n*	264	265	
WHO grade, *n* (%)			0.393
G2	113 (24.2%)	108 (23.1%)	
G3	115 (24.6%)	131 (28.1%)	
IDH status, *n* (%)			<0.001
WT	11 (2.1%)	86 (16.3%)	
Mut	251 (47.7%)	178 (33.8%)	
1p/19q codeletion, *n* (%)			<0.001
Codel	113 (21.4%)	59 (11.2%)	
Noncodel	151 (28.5%)	206 (38.9%)	
Primary therapy outcome, *n* (%)			0.077
PD	45 (9.8%)	65 (14.2%)	
SD	76 (16.6%)	72 (15.7%)	
PR	38 (8.3%)	25 (5.4%)	
CR	73 (15.9%)	65 (14.2%)	
Gender, *n* (%)			0.405
Female	115 (21.7%)	126 (23.8%)	
Male	149 (28.2%)	139 (26.3%)	
Race, *n* (%)			0.653
Asian	4 (0.8%)	4 (0.8%)	
Black or African American	9 (1.7%)	13 (2.5%)	
White	246 (47.5%)	242 (46.7%)	
Age, *n* (%)			0.004
≤40	149 (28.2%)	115 (21.7%)	
>40	115 (21.7%)	150 (28.4%)	
Histological type, *n* (%)			0.002
Astrocytoma	83 (15.7%)	113 (21.4%)	
Oligoastrocytoma	62 (11.7%)	71 (13.4%)	
Oligodendroglioma	119 (22.5%)	81 (15.3%)	
Laterality, *n* (%)			0.320
Left	134 (25.6%)	123 (23.5%)	
Midline	2 (0.4%)	5 (1%)	
Right	124 (23.7%)	136 (26%)	
OS event, *n* (%)			0.003
Alive	212 (40.1%)	182 (34.4%)	
Dead	52 (9.8%)	83 (15.7%)	
DSS event, *n* (%)			0.004
Alive	215 (41.3%)	184 (35.3%)	
Dead	47 (9%)	75 (14.4%)	
PFI event, *n* (%)			0.023
Alive	173 (32.7%)	147 (27.8%)	
Dead	91 (17.2%)	118 (22.3%)	

**Table 4:** Univariate logistic analysis of *hsa-miR-148a-3p* and clinical parameters.

Characteristics	Total (N)	Odds ratio (OR)	*P* value
WHO grade (G3 vs. G2)	467	1.113 (0.774-1.601)	0.565
1p/19q codeletion (noncodel vs. codel)	529	2.712 (1.863-3.983)	<0.001
Primary therapy outcome (PR&CR vs. PD&SD)	459	0.671 (0.462-0.971)	0.035
Age (>40 vs. ≤40)	529	0.948 (0.674-1.334)	0.761
IDH status (Mut vs. WT)	526	0.036 (0.013-0.083)	<0.001
Gender (male vs. female)	529	0.851 (0.604-1.199)	0.357

**Table 5:** Univariate logistic analysis of *hsa-miR-200a-5p* and clinical parameters.

Characteristics	Total (*N*)	Odds ratio (OR)	*P* value
WHO grade (G3 vs. G2)	467	1.192 (0.829-1.716)	0.344
1p/19q codeletion (noncodel vs. codel)	529	2.613 (1.796-3.831)	<0.001
Primary therapy outcome (PR&CR vs. PD&SD)	459	0.716 (0.494-1.036)	0.077
Age (>40 vs. ≤40)	529	1.690 (1.200-2.387)	0.003
IDH status (Mut vs. WT)	526	0.091 (0.045-0.168)	<0.001
Gender (male vs. female)	529	0.851 (0.604-1.199)	0.357

## Data Availability

The authors certify that all the original data in this research could be obtained from public database. miRNA expression data and related clinical factor data of LGG cases were obtained from the TCGA database (https://portal.gdc.cancer.gov/); the immune score of LGG was searched from ESTIMATE (http://bioinformatics.mdanderson.org/estimate/); the target genes of necroptosis-related miRNAs are from TargetScan (http://www.targetscan.org/vert_71/), miRDB (http://mirdb.org/), and miTarBase (http://miRTarBase.cuhk.edu.cn/); the predicted lncRNAs by miRNAs are from starBase (http://starbase.sysu.edu.cn/). And you can contact us for analysis code.
